The article "In Vitro Alpha-Amylase Enzyme Assay of Hydroalcoholic Polyherbal Extract: Proof of Concept for the Development of Polyherbal Teabag Formulation for the Treatment of Diabetes" was published in 2022. Journal: Evid Based Complement Alternat Med.

# *In Vitro* Alpha-Amylase Enzyme Assay of Hydroalcoholic Polyherbal Extract: Proof of Concept for the Development of Polyherbal Teabag Formulation for the Treatment of Diabetes

**DOI:** 10.1155/2022/1577957

**Published:** 2022-05-12

**Authors:** Aamir Quazi, Mohsina Patwekar, Faheem Patwekar, Saad Alghamdi, Bodour S. Rajab, Ahmad O. Babalghith, Fahadul Islam

**Affiliations:** ^1^KT Patil College of Pharmacy, Osmanabad, Maharashtra, India; ^2^Luqman College of Pharmacy, Gulbarga, Karnataka, India; ^3^Department of Pharmaceutical Science, BAMU, Aurangabad, India; ^4^Laboratory Medicine Department, Faculty of Applied Medical Sciences, Umm Al-Qura University, Makkah, Saudi Arabia; ^5^Medical Genetics Department, College of Medicine, Umm Al-Qura University, Makkah, Saudi Arabia; ^6^Department of Pharmacy, Faculty of Allied Health Sciences, Daffodil International University, Dhaka 1207, Bangladesh

## Abstract

For the treatment and maintenance of postprandial blood glucose increases (i.e., diabetes mellitus), alpha (*α*)-amylase is a well-known therapeutic target. In this paper, we report an initial exploration of the work, i.e., *in vitro* alpha-amylase activity of the hydroalcoholic polyherbal extract of the selected plants. After drying, the plant material is ground individually, and at least 100 gm of the crude powder is prepared from each plant. 100 gm of each plant was combined, and a total of 500 gm of the crude powder (*Ichnocarpus frutescens* (100 gm) + *Ficus dalhousie* (100 gm) + *Crateva magna* (100 gm) + *Alpinia galangal* (100 gm) + *Swertia chirata* (100 gm)) was prepared to carry out the extraction. This obtained extract was subjected to preliminary phytochemical screening and *in vitro* alpha-amylase activity. At 16 mg/mL, acarbose displayed 78.40 ± 0.36% inhibition, whereas the extract exhibited 72.96 ± 0.70% inhibition, which is significantly comparable. The IC_50_ value of acarbose was 12.9 ± 1.12, whereas the extract exhibited 13.31 ± 1.12 mg/mL. The extract possesses numerous classes of chemicals such as alkaloids, glycosides, tannins, polyphenols, and terpenoids, which can contribute to the antidiabetic activity through alpha-amylase inhibition. This was an initial exploration of the work as a proof of concept for the development of polyherbal tea bag formulation for the treatment of diabetes. In the future, we are aiming to investigate the effectiveness of polyherbal tea bags in the treatment of diabetes using more *in vitro* and *in vivo* models. From the present investigation, we have concluded that this extract can be used for the treatment of diabetes.

## 1. Introduction

The metabolic disorder known as diabetes mellitus (DM) is characterised by recurrent episodes of high blood sugar. Reduced insulin production, peripheral insulin tolerance, or both may be to blame. The International Diabetes Federation (IDF) estimates that there were around 415 million people aged between 20 and 79 with diabetes mellitus in 2015 [1, 2]. By 2040, there will be an additional 200 million people suffering from DM worldwide. Chronic hyperglycemia and other metabolic abnormalities in patients with diabetes mellitus can harm different organ systems, contributing to the development of life-threatening complications, most of which are microvascular (retinopathy, nephropathy, and neuropathy) and macrovascular complications, which can lead to a 2-fold and 4-fold increased risk of cardiovascular diseases, respectively, in these individuals. Pancreatic beta cells (*β*-cells) generate an insulin hormone that stimulates the absorption of glucose into cells in order to provide energy and is often active in a number of other functions [3, 4]. DM is attributed to a loss of insulin output or insulin sensitivity. It is critical that all types of diabetes should be identified and treated at an early stage to avoid or slow down future problems affecting other organs, such as diabetic nephropathy, retinopathy, neuropathy, cardiovascular disease, and diabetic foot ulcers [5–7].

The article "In Vitro Alpha-Amylase Enzyme Assay of Hydroalcoholic Polyherbal Extract: Proof of Concept for the Development of Polyherbal Teabag Formulation for the Treatment of Diabetes" was published in 2022. Journal: Evid Based Complement Alternat Med.

Diabetes patients throughout the globe are dying and becoming worse at an alarming pace, which necessitates the development of an effective therapy. Because of its effectiveness and safety, traditional medicine is becoming more popular among diabetics. To help with hyperglycemia and muscle versus fat production, herbal treatments may be used. It would be beneficial to do further research on the possible effects of herbal products. If we do frequent item studies on plants, we may find that they have harmful or insufficient effects and illogical outcomes [8, 9]. The greatest antioxidant activity was discovered in a polyherbal mixture of green tea and chosen individual herbs, which had high concentrations of phenolics and flavonoids. Diabetes is better handled by a mixture of herbs (polyherbal) than by a single herb because of synergism and minimal adverse effects in most traditional systems [10–13]. Using a polyherbal composition, a diabetic wound cream was shown to be both efficacious and safe in treating diabetic foot ulcers. Diabetes problems should be prevented as well as managed using an antidiabetic medications therapeutic strategy. Diabetes mellitus may be well managed with normal allopathic treatment, but the results can be restricted. Because of their efficiency in decreasing blood glucose levels and minimal side effects, alternative medicines for diabetes have recently become more popular [11, 14–17]. Alkaloids, flavonoids, and saponins in the plants were responsible for the anticipated therapeutic effect in diabetes mellitus. One plant may contain several phytochemical components; therefore, combining a number of these plants or herbs produces an efficient pharmacological effect. As long as the holistic approach is successful, it may lead to a safer and a more well-tolerated product [18–23].

The article "In Vitro Alpha-Amylase Enzyme Assay of Hydroalcoholic Polyherbal Extract: Proof of Concept for the Development of Polyherbal Teabag Formulation for the Treatment of Diabetes" was published in 2022. Journal: Evid Based Complement Alternat Med.

To form oligosaccharides and monosaccharide glucose, *α*-amylase cleaves the *α*-D-(1,4) glycosidic bonds found in carbohydrates. *α*-Glucosidase then cleaves these oligosaccharides into monosaccharides like glucose. As a result, people who eat a lot of carbohydrate-heavy foods should take inhibitors of these enzymes to keep their blood sugar levels stable [24]. PPHG is now controlled with enzyme inhibitors such as acarbose, miglitol, and voglibose. Only miglitol and voglibose inhibit *α*-glucosidases, but acarbose blocks both *α*-amylase and *α*-glucosidases. They are efficient in reducing PPHG, but the negative effects of these inhibitors make them unsuitable for long-term use [25]. Considering that roughly 80% of diabetics live in poor and middle-income countries, these medicines are incredibly expensive. There have been several attempts to identify *α*-amylase and *α*-glucosidase inhibitors from plants, bacteria, marine algae, and fungus to date. For the most part, scholars have focused on studying crude extracts (organic or aqueous), although a small number have also looked at pure substances themselves. It was shown that the vast majority of plant extracts and pure chemicals were effective against either *α*-amylase or *α*-glucosidase [26, 27].

Phytochemicals derived from plants are currently being employed to treat a wide range of underlying physiological conditions. The potency, purity, and low cost-effectiveness of herbal medicines have made them more popular in recent years. In both traditional and contemporary medicine, plants constitute an important source of bioactive chemicals that contribute to the prevention and treatment of disease. Plant-derived products have long been utilized by people all over the world to treat various ailments [28–30]. After going through the above literature, we have designed a work to formulate a polyherbal teabag for the treatment of diabetes mellitus. For the formulation, we have selected *Ichnocarpus frutescens* [31–33]*, Ficus dalhousiae* [34]*, Crateva magna* [35]*, Alpinia galangal* [36, 37], and *Swertia chirata* [38–41]. All the selected plants have been reported for potential antidiabetic and antioxidant activities. In this paper, we report an initial exploration of the work, i.e., the *in vitro* alpha-amylase activity of the hydroalcoholic polyherbal extract of the selected plants. The hydroalcoholic extract was selected as it extracts the maximum of the phytoconstituents from the plants. The present work aimed to perform a hydroalcoholic Soxhlet extraction of the selected plants by mixing the crude powder of each plant material. The obtained extract was then subjected to the *in vitro* alpha-amylase enzyme assay.

The article "In Vitro Alpha-Amylase Enzyme Assay of Hydroalcoholic Polyherbal Extract: Proof of Concept for the Development of Polyherbal Teabag Formulation for the Treatment of Diabetes" was published in 2022. Journal: Evid Based Complement Alternat Med.

## 2. Materials and Methods

### 2.1. Chemicals and Reagents

Alpha-amylase, 3,5-dinitrosalicylic acid (DNSA reagent), starch, ethanol, conc. hydrochloric acid, sulphuric acid, and different reagents used for qualitative analysis were purchased and procured from Lab Trading Laboratory, Aurangabad, Maharashtra, India. All the chemicals used were of analytical grade.

### 2.2. Collection of Plants and Authentication

The plants *Ichnocarpus frutescens, Ficus dalhousie, Crateva magna, Alpinia galangal*, and *Swertia chirata* were collected and authenticated from Dr. Madhava Chetty, Department of Botany, Sri Venkateswara University, Tirupati, India, with voucher numbers 0448, 0879, 0550, 0911, and 0612 respectively.

### 2.3. Preparation of the Plant Material and Soxhlet Extraction

The collected plants were washed with water to remove any dust or foreign particles present on them and shade-dried for one week at room temperature to avoid excessive loss of volatile phytoconstituents. After drying, the plant material was ground individually, and at least 100 gm of the crude powder was prepared from each plant. 100 gm of each plant was combined, and a total of 500 gm of the crude powder (*Ichnocarpus frutescens* (100 gm) + *Ficus Dalhousie* (100 gm) + *Crateva Magna* (100 gm) + *Alpinia galangal* (100 gm) + *Swertia chirata* (100 gm)) was prepared to carry out the extraction.

The crude powder was subjected to Soxhlet extraction using a hydroalcoholic (30: 70, water: ethanol) solvent. The extraction was carried out till the completion of 10 siphon cycles for at least 48 hours. It was observed that the solvent turned into dark green, ensuring the isolation of maximum phytoconstituents from each plant. The extract was then collected, and the solvent was removed by simple evaporation at room temperature. The crude powder obtained from this process was further utilized for subsequent investigation [42–44].

### 2.4. Pharmacognostical Evaluation and Preliminary Phytochemical Screening of the Extract

#### 2.4.1. Pharmacognostical Evaluation

*(1) Color*. Under direct sunlight, the untreated portion of the medication was taken and its color was observed.

*(2) Odour and Taste*. A little bit of the medication was taken, and the air was breathed slowly and repeatedly over the material to assess the scent of the chemical. To test the taste of the medicine, a little bit of it was put on the tongue.

*(3) Total Ash*. It was necessary to weigh and burn three grams of medication at a temperature not higher than 45 degrees Celsius until the drug was carbon-free and then cool it and weigh it three times until it was stable for three consecutive readings. The air-dried medication was used as a standard to evaluate the ash content.

(1) $$\begin{array}{c} \text{Total ash}=\frac{\text{Wt. of ash}}{\text{Wt. of drug}}\;\times 100. \end{array}$$

*(4) Acid-Insoluble Ash*. It took five minutes of boiling hydrochloric acid to get the whole ash, which was then washed with hot water and burnt to the same weight. The air-dried medication was used as a benchmark to assess the percentage of acid-insoluble ash.

*(5) Alcohol-Soluble Extractive*. A stoppered conical flask was filled with 5 gm of powdered medication and 100 ml of 90 percent alcohol. Using an electric shaker, the flask was shaken constantly for six hours before being allowed to macerate overnight. It was then filtered, and the filter was evaporated to dryness in a subsequent step. The proportion of the extractive was determined by weighing the substance.

(2) $$\begin{array}{c} \text{Alcohol}-\text{soluble extractive}=\frac{\text{Wt. of extractive}}{\text{Wt. of drug}}\;\times 100. \end{array}$$

*(6) Water-Soluble Extractive*. In a stoppered conical flask, 100 ml of chloroform water was added to 5 grams of carefully weighed powdered drug, and the mixture was agitated continually for six hours on an electrical shaker. After maceration, the flask was allowed to sit overnight before being thoroughly filtered and dried using the filter. The proportion of the extractive was determined by weighing the substance [14, 45, 46].

(3) $$\begin{array}{c} \text{Water}-\text{soluble extractive}=\frac{\text{Wt. of extractive}}{\text{Wt. of drug}}\times 100\text{.} \end{array}$$

The article "In Vitro Alpha-Amylase Enzyme Assay of Hydroalcoholic Polyherbal Extract: Proof of Concept for the Development of Polyherbal Teabag Formulation for the Treatment of Diabetes" was published in 2022. Journal: Evid Based Complement Alternat Med.

#### 2.4.2. Preliminary Phytochemical Screening of the Extract

The extract was subjected to preliminary phytochemical screening by various qualitative tests to detect the presence of different classes of phytoconstituents. Different tests such as tests for alkaloids, carbohydrates, steroids, triterpenoids, cardiac glycosides, saponins, tannins, and flavonoids were performed [45, 46].

### 2.5. *In Vitro* Alpha-Amylase Enzyme Assay

In the present evaluation, acarbose was used as control. In a test tube, 1 mL of alpha-amylase and 1 ml of extract were incubated at 37°C for 10 min. After preincubation, each tube was filled with 1 mL of 1% (v/v) starch solution and incubated for 15 minutes at 37°C. The reaction was stopped with 2 mL of DNSA reagent, put in a boiling water bath for 5 minutes, cooled to room temperature, and diluted, and the absorbance was measured using a spectrophotometer at 546 nm (Shimadzu). There was no plant extract in the control process, which represented 100% enzyme activity. The different concentrations of the extract and acarbose were taken (2–16 mg/mL) [27]. The inhibition percentage of alpha-amylase by the extract and acarbose can be calculated:

(4) $$\begin{array}{c} \text{\%inhibition}=\frac{\text{enzyme activity of control}-\text{enzyme activity of extract}}{\text{enzyme activity of control}}\times 100. \end{array}$$

### 2.6. Statistical Analysis

All of the trials were carried out in triplicate. Within the experiments, means, standard errors, and standard deviations were computed from repeated trials. One-way analysis of variance was used for statistical analysis (ANOVA). *P* < 0.05 was considered statistically significant. The GraphPad Prism program was used to determine the IC_50_.

## 3. Results and Discussion

### 3.1. Pharmacognostical Evaluation and Preliminary Phytochemical Screening of the Extract

The yield percent of the extract was found to be 37.89%. The appearance of the extract was dark green, but after drying, a light green powder was obtained with a pungent to bitter odor. The pharmacognostical evaluation of the extract is illustrated in Table 1. The preliminary phytochemical screening results are tabulated in Table 2. From qualitative screening, it was observed that the majority of the phytochemicals were present in the extract.

### 3.2. *In Vitro* Alpha-Amylase Enzyme Assay

The % inhibition with IC_50_ values is tabulated in Table 3. Acarbose was used as control to compare the inhibition effect caused by the extract. The % inhibition caused by the extract in comparison with acarbose is illustrated in Figure 1. The results demonstrated that the extract inhibited the alpha-amylase enzyme significantly and displayed potent activity.

Acarbose is an oral alpha-glucosidase and alpha-amylase inhibitor licensed by the US Food and Drug Administration (USFDA) for the treatment of T2DM. Sugar absorption in the intestine is slowed down and reduced by acarbose, a complex oligosaccharide. This results in a lower postprandial increase in blood glucose levels in T2DM patients. Therefore, in the present study, it was selected as the standard to validate the alpha-amylase activity of the extract [47]. At 16 mg/mL, acarbose displayed 78.40 ± 0.36% inhibition, whereas the extract exhibited 72.96 ± 0.70% inhibition, which is significantly comparable. The extract poses numerous classes of chemicals such as alkaloids, glycosides, tannins, polyphenols, and terpenoids, which can contribute to the antidiabetic activity through alpha-amylase inhibition.

The article "In Vitro Alpha-Amylase Enzyme Assay of Hydroalcoholic Polyherbal Extract: Proof of Concept for the Development of Polyherbal Teabag Formulation for the Treatment of Diabetes" was published in 2022. Journal: Evid Based Complement Alternat Med.

Tea prepared from the leaves, seeds, and/or roots of different plants is known as herbal tea. According to a common belief, they are not generated from the ordinary tea plants, but rather from “tisanes.” Herbal teas have been used for therapeutic purposes for a long time, and there are many different types. Some of them are ingested because of their stimulating effects, which aid in relaxation, digestion control, and immune system strengthening [48]. There are a variety of herbal teas available, including black, green, chamomile, peppermint, ginger, and ginseng. An example is *Astragalus*, a Chinese native plant that has antiinflammatory and antibacterial qualities; in many situations, *Astragalus* tea assists people with HIV and AIDS to manage their symptoms. Drinking herbal tea has been shown to provide several health advantages, with just a few drawbacks [49, 50].

In actuality, herbal teas are more properly referred to as “tisanes,” which are concoctions made from a variety of herbs. It is the mixture of dried leaves, seeds, nuts, and barks, as well as other botanical materials, which give tisanes its flavour and health advantages. Herbal teas, in contrast to most other varieties, do not contain any caffeine. They are also delicious and simple to drink, making them a popular choice. A single herbal component or a combination of herbal ingredients in a herbal tea might be used to achieve a particular goal, including relaxation, rejuvenation, or the alleviation of a certain ailment [51, 52]. Therefore, from the present investigation, we have decided to formulate a polyherbal tea bag containing *Ichnocarpus frutescens, Ficus dalhousiae, Crateva magna, Alpinia galangal*, and *Swertia chirata* extracts. This was an initial exploration of the work as a proof of concept for the development of polyherbal teabag formulation for the treatment of diabetes. In the future, we are aiming to investigate the effectiveness of polyherbal teabags in the treatment of diabetes using more *in vitro* and *in vivo* models.

## 4. Conclusion

There is a broad variety of underlying physiologic problems that may be treated using phytochemicals produced from plants. Herbal medications have grown in popularity in recent years due to their strength, purity, and low cost-effectiveness. Plants are a major source of bioactive compounds that are used in both traditional and modern medicine to prevent and cure illness. People all across the globe have long relied on plant-derived products to cure a wide range of diseases. An enzyme called *α*-amylase breaks down polysaccharide molecules into glucose and maltose, which facilitates digestion. As a result, blood glucose levels and postprandial hyperglycemia increase. Postprandial blood glucose increases may be treated and maintained by targeting *α*-amylase, a well-known enzyme inhibitor. One or more herbal components may be used to make herbal teas, which may then be combined to achieve a particular result, such as relaxation or rejuvenation or relief from a certain ailment. After going through the above literature, we have designed a work to formulate polyherbal tea bag for the treatment of diabetes mellitus. For the formulation, we have selected *Ichnocarpus frutescens, Ficus dalhousiae, Crateva magna, Alpinia galangal*, and *Swertia chirata*, as all the selected plants have been reported for potential antidiabetic and antioxidant activities. At 16 mg/mL, acarbose displayed 78.40 ± 0.36% inhibition, whereas the extract exhibited 72.96 ± 0.70% inhibition which is significantly comparable. As the extract poses numerous class of chemicals such as alkaloids, glycosides, tannins, polyphenols, and terpenoids, it can contribute to the antidiabetic activity through the alpha-amylase inhibition. This was an initial exploration of the work as proof of concept for the development of polyherbal teabag formulation for the treatment of diabetes. In future, we are aiming to investigate the effectiveness of polyherbal teabag in the treatment of diabetes using more *in vitro* and *in vivo* models.

The article "In Vitro Alpha-Amylase Enzyme Assay of Hydroalcoholic Polyherbal Extract: Proof of Concept for the Development of Polyherbal Teabag Formulation for the Treatment of Diabetes" was published in 2022. Journal: Evid Based Complement Alternat Med.

## Figures and Tables

**Figure 1:** The % inhibition caused by the extract in comparison with acarbose at different concentrations.

**Table 1:** The pharmacognostical evaluation of the crude extract.

Parameters	Values (% dry weight basis)
Moisture content	5.7 ± 0.14
Total ash content	6.2 ± 0.17
Water soluble ash content	1.6 ± 0.12
Acid soluble ash content	0.6 ± 0.08
Hot ethanol exactable matter	10.8 ± 0.19
Cold-ethanol extractable matter	8.9 ± 0.21
Hot-water extractable matter	7.7 ± 0.23
Cold-water extractable matter	4.2 ± 0.15

Data are represented as mean ± SEM (standard error mean); *n* = 6.

**Table 2:** The preliminary phytochemical screening of the extract.

Name of chemical class	Polyherbal hydroalcoholic extract
Alkaloid	+++
Carbohydrates	+++
Saponins	+++
Glycoside	+++
Fats and fixed oils	+
Resins	+
Phenols	++
Tannins	+++
Diterpenes	+
Flavonoids	+++
Proteins	++

Here, + indicates present, ++ indicates moderately present, and +++ indicates strongly present.

**Table 3:** The % inhibition of alpha-amylase with IC_50_ values.

Concentrations (mg/mL)	Extract			Acarbose		
	% inhibition	SD	IC_50_ values (mg/mL)	% inhibition	SD	IC_50_ values (mg/mL)
2	11.76	±0.35	13.31 ± 1.12	15.73	±0.40	12.9 ± 1.12
4	16.43	±0.40		20.43	±0.35	
6	21.86	±0.25		25.70	±0.26	
8	27.70	±0.45		32.70	±0.45	
10	36.70	±0.52		42.46	±0.32	
12	48.83	±0.60		53.66	±0.32	
14	60.80	±0.60		68.36	±0.61	
16	72.96	±0.70		78.40	±0.36	

The article "In Vitro Alpha-Amylase Enzyme Assay of Hydroalcoholic Polyherbal Extract: Proof of Concept for the Development of Polyherbal Teabag Formulation for the Treatment of Diabetes" was published in 2022. Journal: Evid Based Complement Alternat Med.

## Data Availability

All data used to support the findings of this study are included within the article.
